The article "SHBG Is an Important Factor in Stemness Induction of Cells by DHT In Vitro and Associated with Poor Clinical Features of Prostate Carcinomas" was retracted in 2020. Reasons: duplicated images; concerns about the data.

# SHBG Is an Important Factor in Stemness Induction of Cells by DHT *In Vitro* and Associated with Poor Clinical Features of Prostate Carcinomas

**DOI:** 10.1371/journal.pone.0070558

**Published:** 2013-07-30

**Authors:** Yuanyuan Ma, Dongming Liang, Jian Liu, Jian-Guo Wen, Einar Servoll, Gudmund Waaler, Thorstein Sæter, Karol Axcrona, Ljiljana Vlatkovic, Ulrika Axcrona, Elisabeth Paus, Yue Yang, Zhiqian Zhang, Gunnar Kvalheim, Jahn M. Nesland, Zhenhe Suo

**Affiliations:** 1 Department of Pathology, The Norwegian Radium Hospital, Institute of Clinical Medicine, Oslo University Hospital, Faculty of Medicine, University of Oslo, Oslo, Norway; 2 Key laboratory of Carcinogenesis and Translational Research (Ministry of Education), Department of Thoracic Surgery II, Peking University Cancer Hospital & Institute, Beijing, China; 3 Department of Surgery, The First Affiliated Hospital of Zhengzhou University, Zhengzhou University, Henan, China; 4 Department of Surgery, Soerlandet Hospital, Arendal, Norway; 5 Departments of Urology, The Norwegian Radium Hospital, Oslo University Hospital, University of Oslo, Oslo, Norway; 6 Department of Medical Biochemistry, Oslo University Hospital, University of Oslo, Oslo, Norway; 7 Key laboratory of Carcinogenesis and Translational Research (Ministry of Education), Department of Cell Biology, Peking University Cancer Hospital & Institute, Beijing, China; 8 Departments of Cell Therapy, The Norwegian Radium Hospital, Oslo University Hospital, University of Oslo, Oslo, Norway; 9 Department of Oncology, The First Affiliated Hospital of Zhengzhou University, Zhengzhou University, Henan, China; Centro de Investigación en Medicina Aplicada (CIMA), Spain

## Abstract

Androgen plays a vital role in prostate cancer development. However, it is not clear whether androgens influence stem-like properties of prostate cancer, a feature important for prostate cancer progression. In this study, we show that upon DHT treatment *in vitro,* prostate cancer cell lines LNCaP and PC-3 were revealed with higher clonogenic potential and higher expression levels of stemness related factors CD44, CD90, Oct3/4 and Nanog. Moreover, sex hormone binding globulin (SHBG) was also simultaneously upregulated in these cells. When the SHBG gene was blocked by SHBG siRNA knock-down, the induction of Oct3/4, Nanog, CD44 and CD90 by DHT was also correspondingly blocked in these cells. Immunohistochemical evaluation of clinical samples disclosed weakly positive, and areas negative for SHBG expression in the benign prostate tissues, while most of the prostate carcinomas were strongly positive for SHBG. In addition, higher levels of SHBG expression were significantly associated with higher Gleason score, more seminal vesicle invasions and lymph node metastases. Collectively, our results show a role of SHBG in upregulating stemness of prostate cancer cells upon DHT exposure *in vitro*, and SHBG expression in prostate cancer samples is significantly associated with poor clinicopathological features, indicating a role of SHBG in prostate cancer progression.

## Introduction

Prostate cancer is a common malignancy in Western countries [1]. Prostate cancer cell growth is initially dependent on androgens. The standard treatment for patients with primary metastatic hormone-dependent prostate cancer is androgen deprivation, and this treatment modality can originally inhibit tumor growth [2], [3]. However, the androgen ablation therapy eventually fails and androgen independent castration resistant prostate cancer (CRPC) develops [4], [5]. The treatment option for metastatic prostate cancer is limited. Metastatic cancer cells are believed to include rare cells that are phenotypically undifferentiated, also called cancer stem cells (CSCs). CSCs are hypothesized to have similar stem cell capacity such as self-renewal, differentiation and initiation of new tumors and are associated with resistance to chemotherapy and radiotherapy [6], [7].

Potent androgens such as testosterone and 5α-dihydrotestosterone (DHT) play an important role in the development of normal prostate and prostate cancer [8], [9]. Testosterone derived in testes is converted to its active form-DHT in the prostate [10]. Androgen receptor (AR) is an androgen-activated transcription factor and a member of the superfamily of nuclear hormone receptors. Sex hormone-binding globulin (SHBG) has also shown a pivotal effect on development of prostate cancers by regulating androgen. SHBG is a 90-kd glycoprotein which is able to bind to sex hormones like testosterone and estradiol, and especially with higher affinity for DHT. In human, SHBG is most expressed in hepatocytes and secreted into plasma [11]. It is also expressed in several other tissues such as testis, breast and prostate which are classic target tissues for androgens and estrogens [12]–[14]. Importantly, SHBG has been demonstrated in tissue sections of human prostate cancers as well as prostate cancer cell lines PC-3, DU145 and LNCaP by immunohistochemistry for protein examination and *in situ* hybridization for SHBG mRNA, suggesting that SHBG is locally regulated and produced [15].

The initial step of androgen and estrogen signaling though SHBG requires binding to its specific receptor (R_SHBG_) on selected cell membranes. Thereafter, subsequent binding of an appropriate androgen or estrogen to the SHBG-R_SHBG_ complex is activated which results in accumulation of cAMP in prostate cancer [16], [17] and breast cancer [18], [19]. Reported downstream effects of SHBG include protein kinase A (PKA) activation [20], induced prostate specific antigen (PSA) expression [21], increased apoptosis [22], and seemingly disparate findings of reduced MCF-7 breast cancer cell growth [23] and increased ALVA-41 prostate cancer cell growth [24].

In this study, we intended to study whether addition of DHT to prostate cancer cell lines LNCaP and PC-3 could influence their stem-like properties. We did observe that upon DHT treatment *in vitro,* prostate cancer cells were revealed with higher clonogenic potential and higher expression levels of stem cell markers CD44, CD90, Oct3/4 and Nanog. In parallel with these findings, the expression of SHBG in these cells was also upregulated after DHT stimulation, and the induction of Oct3/4 and Nanog by DHT was associated with SHBG expression verified by SHBG siRNA knock-down experiments, indicating an important role of SHBG in maintaining cell stemness which may have clinical consequence. Immunohistochemical evaluation of SHBG in clinical samples was then conducted. Weakly positive and areas negative for SHBG expression in the benign prostate tissues was revealed, while most of the prostate carcinomas were strongly positive for SHBG. In addition, the expression of SHBG in the prostate carcinomas was significantly associated with higher Gleason grade score, seminal vesicle invasions and lymph node metastasis.

## Materials and Methods

The ethical committee of the Health Region South-East of Norway has approved this study (REK 2.2007.219). All individuals involved in this project have given written informed consent for the original human work that produced the tissue samples and written informed consent to publish these case details.

### Cell Lines and Cell Treatment

Human prostate cancer cell lines PC-3 and LNCaP were obtained from the American Type Culture Collection (ATCC). All cells were cultivated in RPMI 1640 medium supplemented with 10% fetal bovine serum (FBS) and 100 units/ml penicillin and 100 µg/ml streptomycin in a humidified 5% CO_2_ incubator at 37°C. After allowing cells to attach onto the flasks, the cells were transferred into phenol red-free RPMI 1640 supplemented with 10% charcoal-stripped FBS (androgen-free medium) for overnight. DHT (1 nM or 10 nM; Sigma-Aldrich) was dissolved in ethanol and added in androgen-free medium for cell culture and the corresponding concentration of ethanol was used as blank control [25].

### MTT (3-(4,5-dimethylthiazol-2-yl)-2,5-diphenyltetrazolium Bromide) Assays

PC-3 (1000/well) and LNCaP (2000/well) cells were planted in 96-well plates. After the cells attached to plate, 1 nM or 10 nM DHT was added into the androgen-free medium for variable times. At each time point as indicated, the cells were added with MTT (Sigma-Aldrich) and cultivated at 37°C for 4 hours. Then 200 µL of dimethyl sulfoxide (DMSO, Sigma-Aldrich) was added to each well and mixed thoroughly. The plates were shaken for 15 min and absorbance was determined using spectrophotometer at a wavelength of 570 nm.

### Colony Formation Assay

500/well single cells of PC-3 cells and 1000/well single cells of LNCaP cells were seeded in six-well plates with/without DHT (1 nM or 10 nM) in androgen-free medium as mentioned above for 14 days before the cells were gently washed with PBS and fixed by 4% buffered formalin for 15 min. Subsequently, 1% crystal violet was used to stain the colonies for 30 min. The plates were gently washed with PBS and dried before colony evaluation under microscope. Colony number which contained more than 30 cells was counted and colony formation efficiency was determined as colony formation efficiency = colonies/input cells × 100%.

### Sphere Formation Assay

The sphere assay was performed as described in our previous study [26]. Single PC-3 (500 cells/well) and LNCaP (1000 cells/well) cells were planted in ultralow attachment six-well plates (Ultra low cluster plates, Life sciences). The cells were cultivated in androgen-free medium as mentioned above added with/without DHT (1 nM or 10 nM) for 14 days. More than 30 cells within a sphere was regarded as a full sphere and counted under inverse microscopy. Sphere formation efficiency was determined as following: sphere formation efficiency = sphere/input cells × 100%.

### Flow Cytometry

Based on our previous study [26], the expressions of the surface markers CD44, CD24 and CD90 in the cells treated with/without DHT (10 nM) for 48 hours were analyzed by flow cytometry using a CD44 antibody conjugated with allophycoyanin (APC), a CD24 antibody conjugated with fluorescein isothiocyanate (FITC), and a CD90 antibody conjugated with phycoerythrin (PE). The corresponding APC Mouse IgG2b, FITC Mouse IgG2a, and PE Mouse IgG1 isotype controls were used as negative control and the viable and single cells were gated for analyses on a flow cytometer (Becton Dickinson, San Jose, CA, USA). All the antibodies and isotype controls were obtained from BD Pharmingen.

### Immunoblotting

Cells were washed with ice-cold PBS twice and homogenized in lyses buffer (25 mM Tris HCl pH 7.6, 100 mM NaCl, 1% NP40, 1% Sodium deoxycholate, 0.1% SDS, Thermo Scientific Pierce, Germany) added with protease inhibitors (0.1 uM Aprotinin, 1.0 mM PMSF, 1 uM Leupeptin, 1 uM Pepstatin) immediately before use. The total protein content in samples was measured by the Bio-Rad protein assay (Hercules, CA, USA) according to the manufacturer’s instruction. Equal amounts of protein were resolved by 10% SDS-PAGE and electro-transferred to polyvinylidene difluoride transfer membrane in a Trans-Blot apparatus (Bio-Rad, Hercules, CA). 5% non-fat milk was used to block the membranes and the primary antibodies with optimized concentrations including AR (1 µg/ml), Oct3/4 (2 µg/ml), Nanog (1 µg/ml), SHBG (1 µg/ml) and GAPDH (0.2 µg/m) from R&D system were added to incubate for overnight at 4 °C. The corresponding secondary antibodies conjugated with HRP were then used to incubate the membranes. Immuno-complexes were visualized by enhanced chemiluminescence detection system (GE Healthcare, UK).

### PSA and SHBG Measurements

The PC-3 and LNCaP cells were cultivated in the androgen-free medium added with 1 nM/10 nM DHT for variable periods. Cell culture media at different culture periods were then collected, centrifuged to remove the cellular debris and stored at −70°C for further PSA and SHBG measurement. Total PSA was measured by the time-resolved fluoroimmunometric dual-label assay performed with the AutoDELFIA instrument (AutoDelfia Prostatus PSA Total/Free, Turku, Finland),. The assay was calibrated against WHO standards, with an assay sensitivity of 0.05 ng/ml and interassay coefficient of variation below 5% over the standard range from 0 to 260 ng/ml. The human SHBG ELISA kit (Alpha Diagnostic International, USA) was used for quantitative determination of SHBG in the medium according to the manufacturer’s instruction. A calibrator curve was established and serum positive control was also included for every run.

### Transient Transfection

SHBG siRNA (sc-44847) and siRNA control (sc-33007) for transient transfection were obtained from Santa Cruz Biotechnology. 2×10^5^ cells per well were planted at six-well plates for 24 hours. SHBG siRNA (50 pmols) and siRNA control (50 pmols) were dissolved within OPTI-MEM Reduced Serum Medium and cultivated for 30 min at room temperature separately. Then the transfection mixtures were added onto the 60–80% confluent cells in six-well plates for 5 hours’ cultivation. The medium was aspirated and replaced with fresh normal growth medium for 24 hours. Then the medium was changed to androgen-free medium added with/without DHT (10 nM) for 48 hours. The cells were washed with PBS and harvested for further experiments.

### Clinical Samples

Radical prostatectomy specimens from 117 patients with clinically localized prostate cancer were included in this study. All the patients underwent radical retropubic prostatectomy (RRP) in the period from 1985 until 2006 at Soerlandet County Hospital, Arendal, Norway. The clinical samples were routinely processed for histological diagnosis. Final histological classification in this study was done according to the International Society of Urological Pathology (ISUP, 2005) consensus on Gleason grading of prostate cancer in this study. Gleason grade score, surgical margin (SM) status, seminal vesicle invasion (SVI) and extraprostatic extension (EPE) for the malignant tumors were recorded. In total, five of these patients were found to have lymph node metastasis upon histological re-examination. In addition, formalin-fixed and paraffin-embedded samples from 10 prostate hyperplasia samples were retrieved from the archives of The Norwegian Radium Hospital and included in this study as well.

### Immunocytochemistry and Immunohistochemistry

4µm paraffin sections from paraffin blocks with either cell lines or clinical samples were prepared. After deparaffinization, the sections were treated with hydrogen peroxide (H_2_O_2_) for 5 min to block the endogenous peroxidase. The antibodies for Oct3/4 (AF1759, R&D), Nanog (AF1997, R&D), AR (ABIN165648, DAKO) and two different antibodies for SHBG (CAB-20000TRH, Creative BioMart; AF2656, R&D) were used. The sections were incubated with the primary antibody for 30 min at room temperature. The liver tissue was used as positive control according to the instructions and the non-immune corresponding IgG was used as negative control. After rinsed with DAKO wash buffer, corresponding EnVision FLEX+Linker reagent was added and incubated for 15 min at room temperature before the slides were incubated with the EnVision FLEX+HRP for 30 min at room temperature. The sections were rinsed, colour reaction developed with DAB reagent, counterstained with hematoxylin for 20 seconds, dehydrated and mounted with cover slips before microscopy evaluation. The results were evaluated by two pathologists without knowledge about the patient data. The immunohistochemical results for SHBG for the 117 patients with prostate cancers were assessed according to a previous study [27] as following: 0, no staining like the negative control staining; 1, if a weak positivity was revealed; 2 if a moderate positive staining was observed; and 3 if a strong staining intensity was found. Since only a few carcinomas were either weakly positive or moderately positive, the scores of all the samples were defined as two groups: scores with 1 or 2 were defined as weak expression group, and score 3 was defined as strong expression group.

### Statistical Analyses

All the experiments were performed at least three times. Data are shown as mean ± S.D, Student’s t-test was used to analyze the surface markers expressions and one-way ANOVA was used to assess the cell growth and clonogenicity between different treatments. Comparisons between SHBG expression and clinicopathology variables were analyzed by Pearson chi-square test and Mann-Whitney U test. SPSS software (version 18.0) was used for data analysis and statistical significance was considered as *P*<0.05.

## Results

### Proliferation and Clonogenicity are Stimulated by DHT

Cell growth of prostate cancer cell lines LNCaP and PC-3 treated with two different concentrations (1 nM or 10 nM) of DHT for variable periods of time were examined by MTT assays. Both low and high concentrations of DHT could stimulate the proliferation of androgen-responsive LNCaP cells in both time-dependent and concentration-dependent manners with significantly statistical difference after 48 hours (Figure 1A left panel). The PC-3 cells cultivated with DHT also grew relatively faster than the cell without DHT, although no significant difference was observed in these cells (Figure 1A right panel). We further investigated whether DHT treatment could influence clonogenicity of these two prostate cancer cell lines. As shown in Figure 1B, more clones were demonstrated in cells cultivated with 1 nM DHT and even more clones were observed in both cell lines with 10 nM DHT treatment compared to the control cells without DHT. As also shown in Figure 1C, dose-dependent higher colony formation efficiency was observed in both cell lines. Consistently, DHT treatment could also improve sphere growth for both cell lines, and result in higher sphere formation efficiency for both PC-3 and LNCaP cells in dose -dependent manner as well (Figure 1D and E).

**Figure 1:** DHT induces cell growth and clonogenicity in prostate cancer cell lines. (A) Cell growth curves show statistically significant difference in LNCaP cells with/without DHT treatment, but not in PC-3 cells (* means *P*<0.05). (B) Representative photographs of colony formation in both cell lines demonstrate that more colonies were formed by 1 nM DHT treatment and even more colonies were obtained by 10 nM DHT treatment (bar scale: 50 mm). (C) Histograms of colony formation efficiency show statistically higher efficiencies in the cells treated with low concentration of DHT (*P*<0.01), and even higher efficiencies in the cells by high concentration of DHT (*P*<0.001). (D) Representative photographs for sphere formation for both cell lines in the cells with/without DHT treatment (bar scale: 50 µm). (E) Histograms for sphere formation efficiency show higher efficiencies in the cells added with 1 nM DHT (*P*<0.05), and even higher efficiencies in the cells stimulated with 10 nM DHT (*P*<0.01).

### Stem Cell Surface Markers are Upregulated by DHT

CD44, a candidate stem cell marker for prostate cancer, was upregulated in both prostate cancer cell lines treated with 10 nM DHT for 48 hours, although relatively less prominent in PC-3 cells. As shown in Figure 2A, there was a 1.68-fold increase in CD44 expression in LNCaP cells and 1.22-fold increase in PC-3 cells after DHT treatment. The influence of DHT on the expression of CD24 in these two cell lines was not apparent, with a slightly higher CD24 expression in both cell lines after addition of DHT, with about 1.06-fold increase in LNCaP cells and 1.09-fold increase in PC-3 cells (Figure 2B). Since CD90 has been implicated as a stem cell marker in different studies, we also examined its expression in these cells with/without DHT treatment. As shown in Figure 2C, significantly higher levels of CD90 expression were displayed in both cell lines under DHT treatment (1.81-fold and 1.60-fold increases in LNCaP and PC-3 cells, respectively).

**Figure 2:** Stem-like phenotype analyses by flow cytometry. (A–C) CD44, CD24 and CD90 expressions were analyzed by flow cytometry in LNCaP and PC-3 cells cultivated with/without DHT in 10 nM for 48 hours. CD44 was induced by DHT treatment in both cell lines (A). No statistically significant difference of CD24 expression level was shown in both cell lines (B). CD90 expression was significantly increased by DHT stimulation in both cell lines (C). (* means *P*<0.05).

### The Stemness Factors Oct3/4 and Nanog are Induced upon DHT Treatment

In an attempt to further explore whether stem-like properties of prostate cancer cells were altered in response to DHT, the expressions of stemness factors Oct3/4 and Nanog were investigated in LNCaP and PC-3 cells cultivated with/without DHT for variable periods of time. Both Oct3/4 and Nanog expressions began to be upregulated after 24 hours’ DHT treatment in both cell lines in a concentration-dependent manner (Figure 3A), although Nanog expression was relatively low in comparison to the expression of Oct3/4. The expressions of these two factors were also examined by immunocytochemistry in the cells treated with or without DHT for 48 hours (Figure 3B). In response to DHT treatments, higher levels of Oct3/4 and Nanog expressions were observed in both cell lines. These results were in good agreement with the findings obtained by Western blotting.

**Figure 3:** DHT increases Oct3/4 and Nanog expressions in prostate cancer cell lines. (A) The higher expressions of Oct3/4 and Nanog by immunoblotting assay are shown in LNCaP and PC-3 cells treated with 1 nM and 10 nM DHT treatments, respectively, for variable periods of times. (B) The immunocytochemical staining shows higher levels of these two factors in both cell lines treated with different concentrations of DHT. Human seminoma tissue sections were used as positive controls for these two antibodies (bar scale: 50 µm).

### AR Expression and PSA Secretion are Stimulated by DHT in LNCaP Cells

In consistent with a previous study [28], we also found that AR was positive in LNCaP cells by the methods of Western blotting (Figure 4A left panel) and immnocytochemistry (Figure 4B). The LNCaP cells cultivated in the androgen-free medium showed relatively low level of AR expression and its expression was increased by DHT treatment in both time-dependent and concentration-dependent manners (Figure 4A). Low level of PSA (<5 ng/ml) in LNCaP cells was detected in the androgen-free media. Moreover, there were 4.7-fold and 20.1-fold PSA increases in 24 hours and 48 hours in 1 nM DHT cultivations, respectively, while there were 5.3-fold and 28.4-fold PSA increases in the same time periods in 10 nM DHT cultication in the LNCaP cells (Figure 4A right panel). Immunocytochemistry demonstrated weak nuclear immunostaining for AR in LNCaP cells and stronger expression of this receptor was observed in the cells treated with 1 nM DHT, but strongest AR expression was seen in the cells cultivated with 10 nM DHT (Figure 4B). However, AR was undetectable in PC-3 cells with/without DHT treatment by immunocytochemistry (Figure 4B). In consistent with the negative expression of AR, no PSA was identified by the ELISA assay in the PC-3 cultured media.

**Figure 4:** DHT upregulates AR expression and increases PSA secretion in LNCaP cells. (**A**) DHT upregulates AR expression in LNCaP cells in both time-dependent and concentration-dependent manners (left panel); there are also higher levels of PSA in the DHT treated cells revealed by the ELISA method (right panel). (**B**) Immunocytochemistry shows nuclear positivity of AR in LNCaP cells and its expression is upregulated by DHT treatment; but AR expression is negative in the PC-3 cells with/without DHT treatment (bar scale: 50 µm).

### SHBG is Upregulated by DHT

Since the expressions of Oct3/4 and Nanog could be upregulated in both AR positive LNCaP cells and AR negative PC-3 cells, induction of Oct3/4 and Nanog by DHT through AR was ruled out, at least in the PC-3 cells. Considering the high SHBG affinity to DHT [16], [21], [24], SHBG expression was further examined in LNCaP and PC-3 cells in response to DHT treatment. As shown in Figure 5A, membranous and cytoplasmic SHBG expression was seen in both LNCaP and PC-3 cell lines by immunocytochemistry. Furthermore, 48 hours 1 nM DHT treatment could result in higher levels of SHBG expression, and the highest levels of this protein expression were observed in the cells treated with 10 nM DHT. Western blotting analyses confirmed increased expression of SHBG by DHT treatments in both cell lines (Figure 5A). In parallel with the DHT-induced SHBG expression, Oct3/4 and Nanog expressions were also correspondingly increased by 10 nM DHT treatments in these cells demonstrated by Western blotting.

**Figure 5:** DHT upregulates the expression of stemess factors through SHBG. (A) Stronger immunocytochemical staining of SHBG is shown in LNCaP and PC-3 cells treated with DHT (left panel, bar scale: 50 µm). Immunoblotting demonstrates higher levels of SHBG, Oct3/4 and Nanog expressions in the cells treated with DHT (right panel). (B) SHBG specific siRNA results. SHBG knockdown in both LNCaP and PC-3 cells was verified by immunoblotting (left panel); 10 nM DHT induces expressions of Oct3/4 and Nanog in the cells transfected with the siRNA control, but such an induction disappears in the cells transfected with the specific SHBG siRNA (right panel). (C) LNCaP and PC-3 cells treated with specific SHBG siRNA grow relatively slower compared to the cells cultivated with control siRNA. (* means *P*<0.05). (D) Flowcytometry of CD44 and CD90 (left and right panel, respectively). While 10 nM DHT treatment for 48 hrs induces its expression in both cell lines for both genes (left parts of both panels), there is no CD44 and CD90 expression difference in these cells after specific SHBG siRNA knockdown compared to the siRNA control cells (right parts of both panels).

### Induction of the Stemness Factors is Associated with SHBG Expression

To further investigate whether SHBG was involved in the upregulation of Oct3/4, Nanog, CD44 and CD90 in response to DHT, RNA interference assay was used to suppress endogenous SHBG expression in LNCaP and PC-3 cells. The transient transfection effect was obtained using the siRNA SHBG compared to the siRNA control and the immunoblotting analyses demonstrated that the SHBG-specific siRNA successfully inhibited SHBG expression after transfection for 24 and 48 hours in both cell lines (Figure 5B left panel). Thus, the cells were treated with/without DHT for 48 hours after the cells transfected with siRNA-control or siRNA-SHBG for 24 hours. While higher expressions of Oct3/4 and Nanog was still observed in both LNCaP and PC-3 cells transfected with the siRNA controls and treated with DHT in the cells, the DHT induction of these two factors was blocked in the LNCaP and PC-3 cells treated with the SHBG specific siRNA (Figure 5B right panel), suggesting the induction of these two factors by DHT through SHBG. Relatively slower growth of the LNCaP and PC-3 cells after SHBG knockdown by the specific siRNA was observed, although there was no significant growth difference in the LNCaP cells (Figure 5C). We further examined the effect of SHBG siRNA on the expression of CD44 and CD90 by flowcytometry since their induction was repeatedly observed after DHT treatment. As shown in Figure 5D, no expression induction of CD44 and CD90 could be observed in both cell lines after DHT treatments.

### SHBG is Highly Expressed in Human Prostate Carcinoma

Taking the above results together, greater stem-like properties were displayed by DHT treatment in prostate cancer cell lines and SHBG might play an important role in the induction of stemness features in these cells upon DHT treatment, indicating a potential role of SHBG in prostate carcinomas. To address this question, SHBG expression was investigated in clinical samples including benign and malignant prostate tissues by immunohistochemistry. SHBG expression in liver tissue was always kept as positive control in each running (Figure 6A). Weak and areas negative for SHBG expression were seen in the benign tumor samples. Strong SHBG expression was observed in the prostate carcinomas, especially in the high Gleason grade tumors with highly infiltrating tumor cells (Figure 6B). In the malignant tumors, there were 21 (18%) samples weakly positive, 39 samples (33%) moderately positive, and 57 samples (49%) strong positive for SHBG expression. Typical scores of the prostate carcinomas are shown in Figure 6C.

**Figure 6:** Immunohistochemistry of SHBG expression in prostate cancer tissues. (A) Positive and negative control of SHBG in liver tissues. (B) Weak SHBG positivity is shown in a benign prostate tumor and strong SHBG immunoreactivity is revealed in a malignant Gleason score 8 cancer tissue. (C) Representative immunohistochemical images of different scores of prostate cancer samples are shown. Bar scale in all of the images is 150 µm.

### SHBG Expression is Significantly Associated with Poor Clinicopathological Characteristics

The clinical and pathological characteristics of the 117 patients with prostate cancer are summarized in Table 1. The associations between clinical/pathological features and SHBG expression levels were further analyzed by Pearson chi-square and Mann-Whitney U methods (Table 2). High Gleason grade score for patients with prostate cancer showed a correlation with higher level SHBG expression (*p* = 0.013). It was also found that tumors with higher levels of SHBG expression were more likely to have seminal vesicle invasion compared to the patients with lower level SHBG expression (*p* = 0.017). Importantly, all the tumors with lymph node involvement were shown strong SHBG immunostaining (*p* = 0.009). All the results show that SHBG expression in prostate carcinomas is significantly associated with poor clinicopathological features.

**Table 1:** Clinical and pathologic characteristics for 117 patients with malignant prostate cancer.

Variable:	Median (range) or Frequency (%)
Age:	61 years (44–72)
Preoperative PSA:	7.8 ng/ml (3.4–36.0)
Follow-up:	108 months (14–296)
Gleason score:	
* <7*	34 (29)
* 7a*	48 (41)
* 7b*	18 (15)
* >7*	17 (15)
TNM staging:	
* pT2*	62 (53)
* pT3*	55 (47)

PSA, prostatic specific antigen.

**Table 2:** Comparison of clinical and pathologic characteristics by tumor SHBG intensity.

	SHBG ICH score		p-value
	<3 (weak and moderate)	3 (strong)	
N	60	57	
Age (years)			
≤61	33	26	0.310
>61	27	31	
Preop PSA (ng/ml)			
≤7.8	25	27	0.535
>7.8	35	30	
Gleason score			
<8	56	44	0.013*
8–10	4	13	
UICC staging			
pT2	36	26	0.119
pT3	24	31	
EPE			
−	33	25	0.194
+	26	32	
SVI			
−	57	46	0.017*
+	3	11	
N			
−	48	32	0.009* §
+	0	5	

EPE, extraprostatic extension; SVI, seminal vesicle invasion; N+: lymph node metastases;

* indicates significant difference with *p* value minus 0.05.

§ means 85 patients underwent pelvic lymphadenectomy.

## Discussion

Androgens are essential for prostate cancer development and prolonged administration of testosterone could induce prostate cancer in rodents [29], [30]. Human prostate cancer disease mostly develops into advanced stage-CRPC and even forms metastatic tumors in other organ eventually, although the androgen deprivation treatment is initially effective. Development of CRPC is most probably attributed to cells with stemness features, which endorse the cells with a unique capability in invasion, metastasis and resistance against most of the conventional cancer therapies.

The LNCaP cell line is a human prostate adenocarcinoma cell line derived from lymph node metastasis. This cell line is AR positive. PC-3 is a classical prostatic cell line originally derived from advanced androgen independent bone metastatic prostate cancer. In consistent with the previous study [31], DHT significantly induced proliferation of LNCaP cells. However, we could also see growth stimulation in PC-3 cells, although in a significantly less prominent manner. Due to the notorious association of androgen in prostate carcinogenesis, we attempted to assess whether DHT treatment could influence the stemness features of cells *in vitro*. Indeed, by colony formation and sphere formation assays, both cell lines exhibited a significantly higher colony and sphere formation efficiency, in a dose-dependent manner within the range of 1 nM to 10 nM of DHT. These observations highly indicated an involvement of stemness related molecules.

We further examined the DHT influence on the expressions of CD44, CD24 and CD90 by flow cytometry, since all these molecules have been linked to cells’ stemness. After 48 hours treatment of DHT, significantly higher level of CD44 expression could be repeatedly seen in the LNCaP cells, while the CD44 induction in the PC-3 cells was not the same prominent as in the LNCaP cells, although higher levels of CD44 expression were also observed. This difference may be explained with the fact that PC-3 cells already expressed higher level of CD44 (Figure 2A), and therefore DHT induction of CD44 expression in these cells might be limited. In a previous study, we found that the isolated CD44^bright^ cells of prostate cancer cell lines displayed higher clonogenicity with significantly higher expression levels of stemness-related factors than the corresponding CD44^dim^ cells [26]. The induction of CD44 expression in the current study by DHT is in line with the colony and sphere formation assays. However, CD24 expression in prostate cancer stem cell has been controversial [32], although lack or low expression levels of CD24 were suggested to identify tumor stem cells [33]. We did not find significant difference in CD24 expression in these two cell lines with or without DHT application, indicating that CD24 expression is not associated with cells’ colony formation and sphere formation capability under our experimental condition. CD90, a cell surface molecule, has been identified in a variety of cells including stem and progenitor cells with a function of stemness maintenance [34]–[37]. In good agreement with these findings and our clonogenicity assays, significant increase of CD90 expression was observed in both cell lines upon DHT treatment.

Oct3/4 and Nanog play an important role in maintenance of self-renewal of embryonic stem cell and primordial germ cells. These stemness factors are frequently overexpressed in histologically poorly differentiated tumors than in those well-differentiated tumors [38], an indication that their expressions may be upregulated in the cells with higher stem-like features. Hence we asked whether the expressions of these factors were influenced by DHT. As we expected, significantly higher levels of Oct3/4 and Nanog expressions were found in the DHT treated LNCaP and PC-3 cells in both time and concentration dependent manners, verified by both Western blotting and immunocytochemistry.

All the above results pinpoint to a possibility that DHT indeed upregulates cell stemness of prostate cancer cells *in vitro*. The fundamental biological role of DHT has been characterized via AR. Thus, we further determined to examine the AR status of these two cell lines, in case any AR positivity in the PC-3 cells due to any undiscovered reason or mechanism. However, we verified that the PC-3 cells were still AR negative and not inducible with DHT addition while the LNCaP cells were AR positive and DHT could upregulate the expression of AR in these cells as well, a finding well in line with the previous report (Bonaccorsi et al., 2000). Therefore, we reasoned that it is unlikely the upregulation of the stemness factors Oct3/4, Nanog, CD44 and CD90 in these prostate cancer cell lines was through AR, since similar results were also observed in the AR-negative PC-3 cells. In addition to the genomic action like the classic androgen-AR signaling, a growing body of evidence has suggested that androgen could exert rapid non-genomic effects [39]–[42] such as activated ion channel to increases in free intracellular calcium [43]or sodium [44]. Androgen can stimulate the conventional second messenger signal transduction cascades including PKA, protein kinase C (PKC), and mitogen-activated protein kinases (MAPK) in prostate cancer cells [45]–[47] or in skeletal muscle cells through MAPK pathway [48], [49]. Moreover, androgen binding by SHBG can also stimulate cAMP and PKA in the prostate cancer cell line LNCaP [16], [20]and the SHBG receptor (SHBG-R) could connect to the G protein complex which may conversely bind androgens or influence the activity of a membrane androgen-binding protein indirectly [40]. The fact that the AR negative PC-3 cells responded to DHT treatment with the same stemness upregulation as LNCaP cells rules out the possibility of DHT-AR interaction in stemness maintenance, at least in the PC-3 cells. This encouraged us to explore additional non-genomic molecular association. Since it is known that except AR, DHT has highest binding affinity to SHBG, SHBG should be a molecular candidate to examine in this context. Our results show that SHBG is expressed in both the AR positive LNCaP cells and the AR negative PC-3 cells, verified with both immunocytochemistry and western blotting methods, which are in line with the former report of Hryb et al [15]. Importantly, we found that SHBG was significantly upregulated in both cell lines with DHT stimulation, in parallel with the increasing expressions of Oct3/4, Nanog, CD44 and CD90 upon DHT treatment. However, SHBG secretion was not detectable in the media of LNCaP and PC-3 cells with or without DHT application. This may be due to the sensitivity of the ELISA kit which is usually used for the serum examination of clinical samples with relatively high concentration of SHBG level, or the SHBG expressed in these cells is not secretory. In line with our findings, Loukovaara et al. already reported that 10 nM testosterone and 100 nmol/L to 1 µmol/L cortisol resulted in higher levels of SHBG expression in HepG2 cells, but these treatments did not increase its release into the culture medium, using solid phase two-site fluoroimmunometric assay [50]. The result from Janne’s group also revealed that in the kidney of mice model *shbg* transgene expression is androgen dependent and exogenous androgen increases human SHBG mRNA levels in the kidneys of female mice [51].

Collectively, these results have linked the SHBG expression with cells’ stemness. To further verify this possibility, specific SHBG siRNA was used to suppress endogenous SHBG expression in both cell lines. We have repeatedly demonstrated that when SHBG was blocked down by specific siRNA in these cells, DHT could not upregulate the expressions of the stemness factors Oct3/4, Nanog, CD44 and CD90 in these cells longer, indicating a direct interaction between the induction of these factors by DHT and SHBG. Therefore our results suggest that DHT-SHBG pathway may play an important role in induction of stem-like properties in prostate cancer cells and SHBG expression in prostate cancer samples may be of clinical consequence.

In clinical sample study, all the ten benign prostate tissues were weak and areas negative for SHBG expression. Generally higher levels of SHBG expression were identified in prostate cancer samples compared to the benign prostate tissues. In the prostate carcinomas, infiltrating tumor cells or tumor cells located in the poorly differentiated areas were always strongly positive, while the well-differentiated glandular structures of cancer were always weakly positive for SHBG. Further statistical analyses showed significant association of SHBG with poor pathological characteristics, including high Gleason grade score, involvement of seminal vesicle invasion and lymph node metastasis. In a serum SHBG study, Andrea et al. have also found a similar correlation and suggested that SHBG may be identified as a multivariate predictor of lymph node invasion in prostate cancer patients undergoing extended pelvic lymph node dissection [52]. SHBG in prostate cancer cells is not secretory as we disclosed in our current study. However, it merits further analysis of the mechanism of high levels SHBG in prostate cancer patients as reported by Salonia et al [52].

In conclusion, we have demonstrated that DHT could upregulate prostate cancer cell stemness *in vitro* via SHBG and SHBG expression in prostate carcinomas is significantly associated with higher Gleason grade score, seminal vesicle invasion and lymph node metastasis. All our *in vitro* and clinical sample results indicate an important role of SHBG in prostate cancer progression.
